# Effects of Pramipexole Combined with Nerve Growth Factor on Cognitive Impairment and Urinary AD7c-NTP Expression in Patients with Parkinson's Disease

This article has been retracted.

**DOI:** 10.1155/2022/3398732

**Published:** 2022-04-26

**Authors:** Zhengxin Wang, Saiyu Cheng

**Affiliations:** Department of Neurology and Neurosurgery, The Third Affiliated Hospital of Chongqing Medical University, Chongqing 401120, China

## Abstract

**Objective:**

To explore the effects of pramipexole combined with nerve growth factor (NGF) on cognitive impairment and urinary Alzheimer-associated neural thread protein (AD7c-NTP) expression in patients with Parkinson's disease (PD).

**Methods:**

Fifty patients with PD treated in our hospital from February 2020 to April 2021 were enrolled. The patients were arbitrarily assigned into control group and study group. The former was treated with pramipexole, and the latter was treated with pramipexole combined with NGF. The efficacy, cognitive function, serum inflammatory factors, cortisol levels, serum macrophage migration inhibitory factor (MIF), brain-derived neurotrophic factor (BDNF), urine AD7c-NTP levels, and the incidence of adverse reactions were compared.

**Results:**

First of all, the effective rate in the study group was higher compared to the control group (*P* < 0.05). After treatment, the cognitive function was enhanced, and the scores of Montreal cognitive assessment (MoCA) in the study group were higher compared to the control group (*P* < 0.05). The levels of serum IL-6, CRP, and TNF-*α* decreased after treatment, and the levels of serum IL-6, CRP, and TNF-*α* in the study group were remarkably lower compared to the control group (*P* < 0.05). In addition, the levels of serum DA, NE, and 5-HT increased after treatment, and the levels of serum DA, NE, and 5-HT in the study group were remarkably higher compared to the control group (*P* < 0.05). Then, the levels of serum MIF and urine AD7c-NTP decreased and BDNF increased after treatment, and the level of BDNF in the study group was higher compared to the control group, while the levels of serum MIF and urine AD7c-NTP in the study group were lower compared to the control group (*P* < 0.05). Finally, the adverse reactions were compared. The incidence of adverse reactions in the study group was lower compared to the control group, and the difference exhibited not statistically significant (16.00% vs. 24.00%, *P* > 0.05).

**Conclusion:**

Pramipexole combined with NGF therapy not only can effectively strengthen the cognitive impairment of patients with PD and promote clinical efficacy and high safety but also can inhibit inflammatory state, regulate brain neurotransmitters, and reduce urinary AD7c-NTP levels.

## 1. Introduction

Parkinson's disease (PD) is the most common chronic degenerative disease after Alzheimer's disease (AD), which mainly demonstrates motor symptoms such as ankylosis, bradykinesia, and abnormal posture, as well as nonmotor symptoms (NMS) such as depression, anxiety, hyposmia, and sleep disorder. With the rapid development of global population aging [1]. According to statistics, the prevalence rate of PD over 65 years old in China is 1700/100000, and it increases gradually with the increase of age, and the prevalence rate of male is higher compared to female [2]. The main pathological changes of PD were the degeneration and loss of DArgic neurons in the pars compacta of substantia nigra and the formation of striatum Lewy bodies. At present, the treatment of PD is mainly drug-based symptomatic treatment, and levodopa is the most classic and most frequently used drug. The vast majority of PD patients have remarkably relieved their motor symptoms within 2-5 years after receiving levodopa preparation, but with the use of the drug and the progression of the disease, 70% of 80% of the patients will develop motor complications, including movement fluctuations and dyskinesia, within 5-10 years of use [3]. It has been found that the mechanism of exercise complications may be related to the pharmacokinetics and pharmacodynamics of levodopa, long-term intermittent DA stimulation, and alterations in neurobiochemical metabolism in the brain, such as “pulse” stimulation of DA receptor [3]. Therefore, there is a need to change the type of drug or adjust the dose, such as the use of DArgic receptor (DR) agonists, catechol-O-methyltransferase (COMT) inhibitors, and B-monoamine oxidase (MAO-B) inhibitors, in order to make DA receptor stimulation more sustained. Based on the idea that continuous DA receptor stimulation (CDS) may reduce the incidence of exercise complications, long-acting DA receptor agonists have attracted more attention [4].

PD-related cognitive impairment is one of the most important NMS in patients with PD, which is an independent risk factor impacting the quality of life of patients [5]. PD-related mild cognitive impairment (PD-MCI) is very common in the early stage of PD. Epidemiological investigations have found that about 30% of PD patients can be associated with PD-MCI in the early stage of the disease and may gradually develop into Parkinson's dementia (PDD) increasing the burden of family and social care [5, 6]. At present, PD-MCI markers mainly include imaging, cerebrospinal fluid, blood, urine, and electrophysiological markers, in which imaging, cerebrospinal fluid, and electrophysiological markers have their own advantages and disadvantages [7]. The impairment of white matter function in patients with PD stimulates the material interaction between blood and cerebrospinal fluid, which lays a pathological foundation for the evaluation of PD in urine and blood samples [7, 8]. At present, the research on the related markers of cognitive impairment involves urine AD-associated neurofilament protein (AD7c-NTP) [8]. There are few reports on AD7c-NTP, PD, and PD-MCI at home and abroad. AD7c-NTP is abundant in axons of nerve cells and was first extracted from brain tissue in 1997. At present, AD7c-NTP can be found in cerebral cortex and glial cells of patients with nervous system-related diseases. AD7c-NTP is highly expressed in the frontal and temporal lobes of patients with AD and recognized as a biomarker for early diagnosis of AD [9]. Although AD and PD are two independent diseases, they have overlapping clinical and neuropathological features, so it is speculated that there may be abnormal expression of AD7c-NTP in cerebrospinal fluid or urine of patients with PD, and urine detection of AD7c-NTP is more convenient and noninvasive than cerebrospinal fluid. Therefore, in theory, urinary AD7c-NTP may have an evaluation and early warning effect on cognitive impairment in patients with PD.

Pramipexole is a nonergot dopamine (DA) receptor agonist, which has a high affinity for DA D2 receptor subtypes but has a low affinity for DA D1 receptor, in which the affinity for D3 receptor is 5-7 times higher compared to that for D2 receptor and its affinity to 5-HT2A and 5-HT2B receptors is lower [9]. A study analyzed the plasma concentration of pramipexole sustained-release tablets (4.5 mg/day) and quick-release tablets (1.5 mg). The results demonstrated that the plasma concentration of sustained-release tablets fluctuated less and more stable in 24 hours [10]. A number of studies have found that pramipexole sustained-release tablets can remarkably improve the motor symptoms of early PD patients and delay the use of levodopa [11]. For late PD, in addition to improving motor complications, it can also reduce the dose of levodopa, which can be directly converted from quick-release tablets to sustained-release tablets, most of which do not need dose adjustment [12]. Some studies have suggested that pramipexole and NGF can play a synergistic and complementary effect through different mechanisms to enhance the clinical symptoms of patients with AD who are also patients with neurodegenerative diseases, and the safety performance is worth affirming [13]. The aim of this study is to further verify the effects of pramipexole and NGF on cognitive impairment and urinary AD7c-NTP expression in patients with PD and to provide a clinical prevention and treatment of these diseases as early as possible.

## 2. Patients and Methods

### 2.1. Participant Information

Fifty patients with PD treated in our hospital from February 2020 to April 2021 were enrolled. The patients were arbitrarily assigned into control group and study group. The former was treated with pramipexole, and the latter was treated with pramipexole combined with NGF. In the control group, the age was 43-74 years old, the average age was 65.53 ± 3.55 years, and the course of disease was 0.5-12 years, with an average of 6.24 ± 2.13 years. H-Y grade is as follows: grade 1 in 18 cases, grade 2 in 7 cases, and grade 3 in 5 cases, including 17 males and 18 females. In the study group, the age ranged from 34 to 76 years, with an average of 65.67 ± 3.71 years. The course of disease ranged from 0.5 to 12 years, with an average of 6.64 ± 2.56 years. According to the H-Y grade, there were 15 cases of grade 1, 9 cases of grade 2, and 6 cases of grade 3, including 16 males and 19 females. There was no statistical significance in the general data. This study was permitted by the Medical Ethics Association of our hospital, and written informed consent was obtained from all patients.

Inclusion criteria are the following: (1) primary PD diagnosed according to MDS2015's diagnostic criteria of PD [14]; (2) age 30-80 years old, regardless of gender; (3) “open” stage Hoehn-Yahr grade 1.5-4; (4) patients treated with levodopa plus peripheral decarboxylase inhibitors or other anti-PD drugs (non-DA receptor agonists) have reached a stable dose for at least 30 days; and (5) the patient agreed to receive the research drug treatment, and he or the caregiver could fill in the family diary correctly.

Exclusion criteria are the following: (1) symptomatic or genetically degenerative Parkinson's syndrome; (2) Parkinson's patients with severe dose peak dyskinesia; (3) history of brain stereotactic surgery, nontraumatic rhabdomyolysis, seizures, or drug abuse; (4) suicide attempts or severe suicidal tendencies in the past year (HAMD-17, part III ≥ 5); (5) inability to complete family diaries or poor compliance records; (6) combination of neurotrophic factor, antidepressants, drugs that may cause extrapyramidal adverse reactions or other experimental drugs within 30 days before baseline; (7) pregnant and lactating women; (8) patients with severe renal insufficiency (creatinine clearance < 20 ml/min); (9) other serious systemic or organic diseases, the researchers believe that patients who are unable to evaluate efficacy or are unlikely to complete the expected course of treatment and follow-up (such as malignant tumors and life expectancy < 3 months); and (10) use of DA receptor agonists at least 30 days before baseline.

### 2.2. Treatment Methods

The control group was treated with pramipexole, and the sustained-release tablets of pramipexole hydrochloride were produced by Boehringer Ingelheim Company in Germany, and the specifications were 0.75 mg, respectively. The dose titration method was used at the beginning of administration, and the lowest dose of quick-release tablet (0.375 mg) was given three times a day. After that, increase the dose every 5-7 days, and continue to increase the dose if the patient can tolerate it.

The study group received pramipexole combined with NGF treatment, and the control group received pramipexole with NGF (manufacturer: Lizhu Group Lizhu Pharmaceutical Factory, approval number: S20100005, specification 30 *μ*g) and intramuscular injection, 30 *μ*2 g, qd each time. Both groups were treated continuously for 3 months.

### 2.3. Observation Index

#### 2.3.1. Curative Effect Evaluation

*(1) Clinical Efficacy*. The modified Webster scale was used to evaluate the clinical efficacy, including facial expression, upper limb posture, gait, language, sit-up disorder, and other 10 symptoms. Each symptom was scored by 0-3 points and 4 grades. The higher the score was, the more serious the symptoms were. The decrease rate of total symptom score was taken as the criterion for judging the curative effect. It is effective when the total score decreased ≥60% after treatment; it is effective when the total score decreased ≥30% and<60% after treatment; it is ineffective when the total score decreased <30% or even increased after treatment;treatment effective rate = effective rate + markedly effective rate.

#### 2.3.2. Cognitive Function

*(1) Montreal Cognitive Assessment Scale (MoCA) [15, 16]*. MoCA is an effective tool to evaluate whether patients have mild cognitive impairment in clinic. For the subjects whose educational level is less than 12 years, plus 1 point, the full score is 30, and the score ≥ 26 is normal.

#### 2.3.3. Detection of Serum Inflammatory Factors

*(1) Serum Inflammatory Factors*. Before treatment and 3 months after treatment, fasting venous blood 4 ml was collected, and serum was collected to detect the contents of serum interleukin-6 (IL-6), C-reactive protein (CRP), and tumor necrosis factor-*α* (TNF-*α*) by enzyme-linked immunosorbent assay (ELISA).

#### 2.3.4. Detection of Brain Neurotransmitter Level

*(1) Brain Neurotransmitters*. Before treatment and 3 months after treatment, the contents of brain neurotransmitters such as dopamine (DA), norepinephrine (NE), and 5-hydroxytryptamine (5-HT) were measured by ML2001 EEG ultraslow fluctuation analyzer of Beijing Tongren Optoelectronic Technology Company.

#### 2.3.5. Serum MIF, AD7c-NTP, and BDNF Horizontal Detection

Detection of serum macrophage cytokines: the fasting elbow venous blood of all subjects was collected for 5 ml, and the samples were placed in a non-anticoagulant test tube and placed at room temperature, then centrifuged with 3000 r/min for 15 minutes with a centrifugal radius of 16 cm. The serum was taken after centrifugation and stored in the refrigerator at 80 ℃. Then the macrophage factors in the serum were detected by enzyme-linked immunosorbent assay (kit purchased from Hangzhou Novak Biotechnology Co., Ltd., batch number 2017103081).. Urine AD7c-NTP was detected, and urine 20 ml was taken from all subjects in the morning, and urine AD7c-NTP was detected by enzyme-linked immunosorbent assay (kit purchased from Shanghai JJ7091412). The operation was completed in strict accordance with the reagent instructions. BDNF was detected. Fasting venous blood 4 ml was taken from all subjects at about 10: 00 in the morning. The supernatant was separated and stored at 80°C. The level of BDNF was examined by enzyme-linked immunosorbent assay (kit purchased from Sambega (Nanjing) Biological Company; production batch number J2017050712), and the level of serum BDNF was detected according to the reagent manual.

#### 2.3.6. Incidence of Adverse Reactions

The incidence of adverse reactions was calculated.

### 2.4. Statistical Analysis

SPSS 21.0 software was employed for statistical analysis, *t*-test was employed for comparison of measurement data, and rank sum test was employed for measurement data of nonnormal distribution, which was presented by mean ± standard deviation ($\bar{x}\pm \text{s}$). The counting data were compared by *χ*^2^ or Fisher's exact probability method. *P* < 0.05 indicated that the difference exhibit statistically significant, and *P* value less than 0.001 was viewed as highly statistically significant.

## 3. Results

### 3.1. Comparison of Clinical Efficacy

First of all, we compared the clinical efficacy: the study group was remarkably effective in 13 cases, effective in 11 cases, and ineffective in 1 case, and the effective rate was 96.00%; the control group was remarkably effective in 8 cases, effective in 11 cases, and ineffective in 6 cases, and the effective rate was 76.00%. The effective rate in the study group was higher compared to the control group (*P* < 0.05). All the results are indicated in Figure 1.

### 3.2. Comparison of Cognitive Function Scores

Secondly, we compared the cognitive function, and there was no significant difference before treatment, but after treatment, the cognitive function was enhanced, and the scores of MoCA in the study group were higher compared to the control group (*P* < 0.001). All the results are indicated in Table 1.

### 3.3. Comparison of the Levels of Serum Inflammatory Factors

Thirdly, we compared the levels of serum inflammatory factors, and there was no significant difference before treatment, but after treatment, the levels of serum IL-6, CRP, and TNF-*α* decreased, and the levels of serum IL-6, CRP, and TNF-*α* in the study group were lower compared to the control group (*P* < 0.001). All the results are indicated in Table 2.

### 3.4. Comparison of the Changes of Brain Neurotransmitters

Then, we compared the levels of serum cerebral cortisol, and there was no significant difference before treatment, but after treatment, the levels of serum DA, norepinephrine (NE), and 5-hydroxytryptamine (5-HT) increased, and the levels of serum DA, NE, and 5-HT in the study group were remarkably higher compared to the control group (*P* < 0.001). All the results are indicated in Table 3.

### 3.5. Serum MIF, BDNF, and Urine AD7c-NTP Horizontal Contrast

Next, we compared the levels of serum MIF, BDNF, and urinary AD7c-NTP, and there exhibited no significant difference before treatment. After treatment, the levels of serum MIF and urinary AD7c-NTP decreased and BDNF increased, and the level of BDNF in the study group was higher compared to the control group, while the levels of serum MIF and urine AD7c-NTP in the study group were lower compared to the control group (*P* < 0.001). The results are indicated in Table 4.

### 3.6. Comparison of Adverse Reactions

Finally, the adverse reactions were compared. There were no serious adverse reactions; there were 2 cases of nausea, 2 cases of vomiting, and 2 cases of diarrhea in the control group and 1 case of nausea, 1 case of vomiting, 1 case of diarrhea, and 1 case of anorexia in the study group. The incidence of adverse reactions in the study group was lower compared to the control group, and the difference exhibited not statistically significant (16.00% vs. 24.00%) (*P* > 0.05). All the results are indicated in Figure 2.

## 4. Discussion

PD is very common in the degenerative diseases of the nervous system, and the middle-aged and elderly people have a high incidence of PD [12]. The typical clinical manifestations of PD are tremor, rigidity, dyskinesia, posture maintenance, and balance disturbance [13]. Meanwhile, some NMS are also common in most PD patients, such as anxiety, depression, loss of smell, constipation, and restless leg syndrome [14]. Cognitive impairment is the most frequent form of NMS in patients with PD, but considering that the early cognitive impairment in most patients is mild and not prominent, we cannot find and pay attention to it early in clinic [17]. According to the reports of the Oxford PD Center, almost all cognitive performance in the PD group decreased remarkably compared with the normal group, including memory, computing power, attention, visual space, executive function, and thinking agility as the main typical manifestations [15]. Clinically, DA replacement therapy has become the main treatment of PD. However, the response to DA varies from person to person. DA cannot relieve all the clinical symptoms of patients with PD, nor can they change the progression of the disease [16]. On the contrary, excessive DA supplementation can also cause cognitive impairment [18]. Some researchers have found that about half of the patients with PD would have clinical manifestations such as decreased memory, visual space, and executive function, thus further developing into dementia (PDD) [19]. Before PD patients develop into PDD, there will also be cognitive impairment in a transitional period, which is called PD mild cognitive impairment (PD-MCI). With regard to the guidelines for the diagnosis of PD with cognitive function [20], the International Dyskinesia Association proposes that patients with PD can be diagnosed if there is clear evidence of cognitive impairment through neuropsychological scale and cognitive function scale test. In all patients with PD, we found that PD-MCI can be present in both early and late stages of PD.

Levodopa has always been considered to be the most classical and effective treatment for PD, which can remarkably improve patients' symptoms within several years of initial treatment [21]. However, with the gradual progress of PD, it is necessary to increase the dose of levodopa to enhance the symptoms and quality of life. Furthermore, 7-8 years after the treatment of levodopa, the curative effect will decrease and exercise complications will occur, which will critically affect the quality of life of patients, while delayed, low-dose levodopa use can reduce the risk of exercise complications [22]. Therefore, drugs that can replace levodopa, delay the use of levodopa, and reduce the dose of levodopa have become the latest choice for patients with PD. Pramipexole is a nonergot DA receptor agonist, which selectively binds to the DA D2 receptor family and has a high affinity for D3 receptors in this family. Studies have indicated that pramipexole can protect nerve cells from apoptosis induced by MPP+, inhibit and reduce the damage of quinones to substantia nigra cells, and then reduce the adverse reactions caused by long-term use of levodopa [21]. The comparison of blood concentration demonstrates that the fluctuation of blood concentration of ER is smaller compared to IR, and there is no peak of drug concentration caused by repeated use [22]. To the maximum extent, it achieves “continuous” DA receptor stimulation and follows the important principle of combining symptom improvement with prevention and treatment of long-term complications in the selection of anti-PD drugs. In addition, taking it once a day also greatly facilitates PD patients who often need to combine several drugs and improves their compliance [22].

NGF is the earliest and most thoroughly studied neurotrophic factor, which has the dual biological functions of neuron nutrition and promoting neurite growth [23]. NGF plays a key role in regulating the development, differentiation, growth, regeneration, and expression of functional characteristics of central and surrounding neurons. The dimer composed of two 118 amino acids through noncovalent bond is highly homologous to the structure of human NGF, and the biological effect has no obvious interspecific specificity [23]. When the effector neurons of NGF are damaged, such as axotomy, drug damage, or even ischemia or hypoxia, a series of pathological changes will occur, including death. Experimental studies have confirmed that NGF can remarkably reduce or prevent the secondary pathological damage by inhibiting the release of toxic amino acids, calcium overload, release of superoxide free radicals, and apoptosis [23].

Combined with the results of this study, compared with the clinical efficacy of the two groups, the effective rate of the study group was higher compared to the control group (*P* < 0.05). After treatment, the cognitive function was enhanced. The scores of MoCA in the study group were higher compared to the control group, and the difference exhibited statistically significant. The levels of serum IL-6, CRP, and TNF-*α* decreased after treatment, and the levels of serum IL-6, CRP, and TNF-*α* in the study group were remarkably lower compared to the control group. And the levels of serum DA, NE, and 5-HT increased after treatment, and the levels of serum DA, NE, and 5-HT in the study group were remarkably higher compared to the control group. The analysis demonstrated that the main pathological alterations of PD were degeneration and necrosis of DArgic neurons in the dense part of substantia nigra, decrease of DA content in striatum, Lewy bodies in the cytoplasm of residual neurons in substantia nigra, and acetylcholine hyperactivity, which led to the decrease of brain tissue content. The death rate of DA neurons in substantia nigra is more than 50%, the content of DA in striatum is reduced by more than 80%, and the content of acetylcholine is reduced by more than 70% [24]. The principle of clinical treatment is to select appropriate drugs to inhibit the activity of acetylcholine in the brain and increase the content of DA. NGF is an important bioactive molecule in the nervous system, which can promote the development of peripheral and central neurons and inhibit the continuous damage of neurons in patients with PD. Pramipexole can directly activate the postsynaptic membrane DA receptor in the absence of DA, so as to enhance clinical symptoms. The combination of the two can effectively facilitate the cognitive impairment of PD patients, enhance the clinical treatment effect, and strengthen the treatment safety.

AD7c-NTP is a transmembrane phosphoprotein produced by neurons, located in neuronal axons, and is widely present and selectively overexpressed in neurofibrillary tangles (NFTs) in the brain of patients with AD. At present, AD7c-NTP has become one of the important biomarkers for predicting AD [25]. Some scholars have confirmed that the overexpression of AD7c-NTP induced by isopropyl-*β*-D-thiogalactoside (IPTG) can lead to neuronal degeneration and apoptosis, damage of mitochondrial function, and other changes similar to those of neurons in patients with AD, suggesting that AD7c-NTP is closely related to neuronal damage in the brain of patients with AD [26]. Some scholars have found that the abnormal expression of AD7c-NTP can early predict the occurrence of degenerative events of neurodegenerative diseases [27]. Further studies confirmed that increased levels of AD7c-NTP could be detected in brain tissue extract, cerebrospinal fluid, and urine of patients with MCI and AD, and the degree was positively correlated with the severity of cognitive impairment [28]. Regarding the recognized biomarkers of AD, AD7c-NTP can be detected from cerebrospinal fluid and urine at the beginning of neuronal degeneration. Additionally, urine samples are more convenient, so urinary AD7c-NTP has become an effective index for the diagnosis of early cognitive dysfunction. The current study found that urinary AD7c-NTP levels were increased in patients with 48.60% MCI in AD patients and normal in 90.70% nondementia patients, suggesting that urinary AD7c-NTP is a high-risk factor for cognitive impairment [29]. At present, it has been confirmed that the expression level of AD7c-NTP in cerebrospinal fluid and brain tissue of patients with neurodegeneration is selectively increased. In recent years, urinary AD7c-NTP has been widely employed in the study of neurodegenerative diseases outside AD.

Of note, the study reported that 80% of PD patients were complicated with cognitive impairment, and 30% of patients developed Parkinson's dementia. Some studies have found that the occurrence of dementia in patients with PD is not only related to cognitive impairment but also related to serum inflammatory factors [30]. Serum MIF is a marker of slow and acute inflammation, which can promote the development of PD. BDNF is an important neurotrophic factor in the brain. And studies have indicated that it cannot only repair cerebral ischemic injury but also attaches importance in learning and memory [31]. Other studies have found that the level of urinary AD7c-NTP in patients with cognitive impairment is remarkably higher compared to normal people, and it is considered that its level is related to the severity of the patient's condition [31]. MIF, BDNF, and urinary AD7c-NTP are closely related to cognition, but there are few reports on whether the levels of MIF, BDNF, and urinary AD7c-NTP are related to cognitive impairment in patients with PD. In this study, after treatment, the levels of serum MIF and urine AD7c-NTP decreased and BDNF increased, and the level of BDNF in the study group was higher compared to the control group, while the levels of serum MIF and urine AD7c-NTP in the study group were lower compared to the control group. The analysis demonstrated that MIF was a marker of serum acute and chronic inflammation, and the level of serum MIF was remarkably increased in patients with inflammatory reaction, and it was more sensitive than CRP in judging the degree of acute and chronic inflammatory reaction. Some scholars have conducted studies on patients with PD and dementia and found that the level of serum MIF is increased, and intervention on inflammatory reaction found that it can improve the motor dysfunction of the patients [32]. Serum MIF can block the extracellular signal-regulated kinase signal pathway, reduce the protection of microglia, and increase nerve damage. It also demonstrates that the degree of microglia damage is related to the severity of inflammation and symptoms. Based on the study of neuroinflammation in patients with PD, it is found that neuroimmune mediated by microglia in the brain leads to nerve cell damage and cognitive impairment. The study also found that the selective increase of AD7c-NTP expression in the urine of patients with cognitive impairment was related to neurodegeneration. Some studies have compared the urinary AD7c-NTP levels between patients with cognitive impairment of AD and normal people [33]. The results show that after receiving pramipexole combined with NGF treatment, the cognitive function of patients in the study group is remarkably enhanced, and the level of urinary AD7c-NTP is also remarkably decreased. A large number of studies have demonstrated that when neurons are damaged, BDNF binds to its receptors, using antioxidant, antiapoptosis, and other mechanisms to prolong the survival time of neurons, so as to play its protective role. With the deeper research, it has been found that serum BDNF not only plays a key role in repairing brain injury but also plays a key role in human memory and learning. Scientific studies have pointed out that BDNF attaches importance in the formation and enhancement of human memory, the expression of BDNF mRNA increases, and the activity of its high affinity receptor factor increases remarkably [34].

Taken together, pramipexole combined with NGF therapy not only can effectively strengthen the cognitive impairment of PD patients and enhance clinical efficacy and high safety but also can inhibit inflammatory state, regulate brain neurotransmitters, and reduce urinary AD7c-NTP levels.

## Figures and Tables

**Figure 1:** Comparison of curative effect between two groups.

**Figure 2:** Comparison of incidence of adverse reactions between two groups.

**Table 1:** Comparison of MoCA scores between the two groups ($\bar{x}\pm \text{s}$, points).

Group	*N*	MoCA scoring	
		Before treatment	After treatment
C group	25	21.84 ± 1.33	22.68 ± 1.22
R group	25	21.69 ± 1.35	25.23 ± 2.31
*t*		0.395	4.880
*P*		0.694	<0.001

**Table 2:** Comparison of serum inflammatory factors between the two groups [$\bar{x}\pm \text{s}$].

Group	*N*	IL-6 (pg·ml^−1^)		CRP (mg·L^−1^)		TNF-*α* (pg·ml^−1^)	
		Before treatment	After treatment	Before treatment	After treatment	Before treatment	After treatment
C group	25	220.86 ± 32.55	169.93 ± 26.32	3.49 ± 0.45	2.25 ± 0.23	2.94 ± 0.34	2.31 ± 0.32
R group	25	220.38 ± 31.67	132.75 ± 22.67	3.48 ± 0.39	1.39 ± 0.21	2.98 ± 0.32	1.38 ± 0.16
*t*		0.052	5.351	0.083	13.806	0.428	12.997
*P*		0.958	<0.001	0.933	<0.001	0.670	<0.001

**Table 3:** Comparison of cerebral cortisol levels between the two groups [$\bar{x}\pm \text{s}$].

Group	*N*	DA		NE		5-HT	
		Before treatment	After treatment	Before treatment	After treatment	Before treatment	After treatment
C group	25	3.78 ± 0.66	6.68 ± 0.64	9.83 ± 1.04	12.18 ± 1.75	18.94 ± 2.15	21.84 ± 2.67
R group	25	3.79 ± 0.67	8.83 ± 1.84	9.89 ± 1.08	14.58 ± 1.35	18.98 ± 2.46	24.68 ± 3.33
*t*		0.053	5.518	0.200	5.429	0.061	3.326
*P*		0.957	<0.001	0.842	<0.001	0.951	0.001

**Table 4:** Serum of patients in two groups MIF, BDNF, and urine AD7c-NTP horizontal contrast [$\bar{x}\pm \text{s}$].

Group	*N*	MIF (*μ*mmol/l)		BDNF (ng/ml)		Urine AD7c-NTP (ng/ml)	
		Before treatment	After treatment	Before treatment	After treatment	Before treatment	After treatment
C group	25	45.84 ± 3.31	37.42 ± 2.44	4.81 ± 2.16	7.85 ± 2.47	5.83 ± 1.64	3.95 ± 1.54
R group	25	45.81 ± 3.44	32.59 ± 2.34	4.89 ± 2.45	11.82 ± 2.44	5.89 ± 1.45	2.55 ± 1.44
*t*		0.031	7.143	0.122	5.717	0.137	3.320
*P*		0.975	<0.001	0.903	<0.001	0.891	<0.001

## Data Availability

No data were used to support this study.

## References

[1] Xing C., Fengbo X., Tingting L. (2021). Correlation analysis of olfactory function, cognitive function and motor symptoms in patients with PD. *Chinese Journal of Modern Neurological Diseases*.

[2] Ma Q., Yang R., Xinyi O., Zhou D. (2021). Clinical effect of Buzhong Yiqi decoction combined with domperidone on patients with PD with delayed gastric emptying and weakness of spleen and stomach. *Proprietary Chinese Medicine*.

[3] Giuseppe A., Nazanine M., Rejko K. (2021). Exploring the contribution of the mitochondrial disulfide relay system to PD: the PINK1/CHCHD4 interplay. *Neural Regeneration Research*.

[4] Carla F., Joana C., Sandra T., Quintas A. (2021). A biophysical perspective on the unexplored mechanisms driving PD by amphetamine-like stimulants. *Neural Regeneration Research*.

[5] Jie Z., Manish K., Jeevan S., Yuan Z. (2021). Arbutin effectively ameliorates the symptoms of PD: the role of adenosine receptors and cyclic adenosine monophosphate. *Neural Regeneration Research*.

[6] He L., You Q., Chen G. (2021). Effect of estradiol on Cav 1.3 gene expression in PC12 cells in PD cell injury model. *Chinese Journal of Gerontology*.

[7] Chao J. Y., Xiong K. P., Zhuang S. (2021). Relationship between emotional apathy and motor symptoms, sleep and cognitive function in patients with early PD. *Chinese Medical Journal*.

[8] Wu M., Qinglun S., Zhenjie S. (2021). Effects of paeoniflorin activated autophagy on motor ability and DArgic neurons in mice with PD. *Chinese Journal of Neuromedicine*.

[9] Lu M., Peng F., Guo Y., Cheng H., Guofang X. (2021). Effects and mechanism of a novel enterotropic insulin double receptor agonist on gait behavior in mice with subacute PD. *Chinese Journal of Geriatric Cardiovascular and Cerebrovascular Diseases*.

[10] Jiecheng F., Wang J., Chunfeng X., Liu S., Guo P., Shuyun Z. (2021). Effects of respiratory function training on motor and respiratory function and activities of daily living in patients with PD. *Chinese Journal of Physical Medicine and Rehabilitation*.

[11] Camilla R., Rocco C., Matteo C. (2021). Sudomotor and cardiovascular autonomic function in de novo PD assessed by sudoscan and cardiovascular reflexes. *Journal of the Neurological Sciences*.

[12] Yang G., Wu M., Mengmeng Q., Jiao J. (2021). Diagnostic value of P 300 combined with MoCA in patients with PD. *Chinese Journal of Gerontology*.

[13] Yu Z. L., Jin Q.-Q., Hölscher C., Li L. (2021). Glucagon-like peptide-1/glucose-dependent insulinotropic polypeptide dual receptor agonist DA-CH5 is superior to exendin-4 in protecting neurons in the 6-hydroxy DA rat Parkinson model. *Neural Regeneration Research*.

[14] Ricardo M., Francisco O., Fradique M. (2021). Automatic classification of idiopathic Parkinson’s disease and atypical Parkinsonian syndromes combining [11C] raclopride PET uptake and MRI grey matter morphometry. *Journal of Neural Engineering*.

[15] Huifang S., Wang Z., Qi Z. (2021). Generation of induced pluripotent stem cell line (ZZUi027-a) derived from skin fibroblasts from a PD patient with RAB39B gene mutation. *Stem Cell Research*.

[16] Sharp ME., Duncan K., Foerde K., Shohamy D. (2020). Dopamine is associated with prioritization of reward-associated memories in Parkinson's disease. *Brain*.

[17] Javier P., Michele T., Carla C., Jost W. H. (2021). The role of glutamatergic neurotransmission in the motor and NMS in PD: clinical cases and a review of the literature. *Journal of Clinical Neuroscience*.

[18] Qiwen H., Tan F., Yali L., Haiqiao W. (2021). Effect of high frequency repetitive transcranial magnetic stimulation combined with neuromuscular stimulation on UPDRS motor score in elderly patients with PD. *Chinese Journal of Gerontology*.

[19] Jonas G., Lynn V., Frédéric M. (2021). Influence of probiotic bacteria on gut microbiota composition and gut wall function in an in-vitro model in patients with PD. *International Journal of Pharmaceutics: X*.

[20] Fahd B., Mihaela B., Lucy M. (2021). Per-oral image guided gastrojejunostomy insertion for levodopa-carbidopa intestinal gel in PD is safe and may be advantageous. *Parkinsonism and Related Disorders*.

[21] Wang W., Ziyan L., Gao J. (2021). Treadmill exercise alleviates neuronal damage by suppressing NLRP3 inflammasome and microglial activation in the MPTP mouse model of PD. *Brain Research Bulletin*.

[22] Andrea R., An V., Schindlbeck K. A. (2021). PD-related pattern (PDRP) identified using resting-state functional MRI: validation study. *Neuroimage: Reports*.

[23] Malin P., Anders B., Tomas B. (2021). In vivo conversion of DA neurons in mouse models of PD — a future approach for regenerative therapy?. *Current Opinion in Genetics & Development*.

[24] Dejan G., Maruša M., Robert R. (2021). Long-term effect of bilateral STN-DBS on NMS in PD: a four-year observational, prospective study. *Parkinsonism & Related Disorders*.

[25] Xiumin L., Weiwei L., Wang C. (2021). Silibinin attenuates motor dysfunction in a mouse model of PD by suppression of oxidative stress and neuroinflammation along with promotion of mitophagy. *Physiology & amp; Behavior*.

[26] Ning L., Yi L., Yali Q., Cheng H., Yan C., He W. (2021). Study on network pharmacology and molecular docking of Rehmannia glutinosa Yinzi in treating AD and PD. *Chinese Journal of Traditional Chinese Medicine Information*.

[27] Chandra T. U., Punna R. R., Dalvi Avantika V. (2021). Design, optimization and pharmacokinetic evaluation of piribedil loaded solid lipid nanoparticles dispersed in nasal in situ gelling system for effective management of PD. *International Journal of Pharmaceutics*.

[28] Hideaki N., Arisa K., Shuji W., Honjoh K., Matsumine A. (2021). Clinical and imaging features of surgically treated low lumbar osteoporotic vertebral collapse in patients with PD. *Scientific Reports*.

[29] Ji F., Zhuo L., Fang W., Yu K. (2021). Prevalence of malnutrition/malnutrition risk and nutrition-related risk factors among patients with PD: systematic review and meta-analysis. *Nutritional Neuroscience*.

[30] Gonzalez-Latapi P., Bayram E., Litvan I., Marras C. (2021). Cognitive impairment in Parkinson's disease: epidemiology, clinical profile, protective and risk factors. *Behavioral Sciences*.

[31] Zhu C., Bilousova T., Focht S. (2021). Correction to: Pharmacological inhibition of nSMase2 reduces brain exosome release and *α*-synuclein pathology in a PD model. *Molecular Brain*.

[32] Rocha N. P., de Miranda A. S., Teixeira A. L. (2015). Insights into neuroinflammation in Parkinson's disease: from biomarkers to anti-inflammatory based therapies. *BioMed Research International*.

[33] Zhang Y., Li Y., Wang R., Sha G., Jin H., Ma L. (2020). Elevated urinary AD7c-NTP levels in older adults with hypertension and cognitive impairment. *Journal of Alzheimer's Disease*.

[34] Hoon L. J., JiHye H., Hye J. E., Jou I. (2021). Small heterodimer partner (SHP) aggravates ER stress in PD-linked LRRK2 mutant astrocyte by regulating XBP1 SUMOylation. *Journal of Biomedical Science*.

